The article "Upregulating hsa-miR-128a Increased the Effects of Pembrolizumab on Laryngeal Cancer Cells via the p53 Pathway" was retracted in 2024. Reasons: signs of a paper mill; unreliable results or conclusions; concerns about the results or conclusions; concerns about the peer review.

# Upregulating hsa-miR-128a Increased the Effects of Pembrolizumab on Laryngeal Cancer Cells via the p53 Pathway

**DOI:** 10.1155/2021/2342784

**Published:** 2021-03-18

**Authors:** Hui Chen, Yang Guo, Jiameng Huang, Liang Zhou

**Affiliations:** Department of Otolaryngology-Head and Neck Surgery, Eye and ENT Hospital of Fudan University, No. 83, Fenyang Road, Xuhui District, 200031 Shanghai, China

## Abstract

**Objectives:**

Recently, immunotherapy and microRNA have shown much more promises in oncology research, inspiring new hope for a cure for various malignancies. Specifically, the function and mechanisms of action of pembrolizumab have been investigated in many cancers, but not in laryngeal squamous cell carcinoma. The present study thus focused on the effect of hsa-miR-128a on pembrolizumab in laryngeal cancer cells as well as tried to elucidate the mechanisms that may mediate this effect.

**Methods:**

Hep2 and AMC-HN8 cell lines were utilized to create stable cell lines that overexpressing hsa-miR-128a. Using the immunotherapy assay, the contribution of hsa-miR-128a to pembrolizumab sensitivity was evaluated. By performing the dual luciferase assay and quantitative real-time polymerase chain reaction, the possible mechanisms of hsa-miR-128a were identified.

**Results:**

Hsa-miR-128a was overexpressed in laryngeal cancer cell lines successfully. The immunotherapy assay revealed that upregulating hsa-miR-128a augmented the effect of pembrolizumab. Moreover, hsa-miR-128a targeted BMI-1 and might played a role in the p53 pathway.

**Conclusion:**

Hsa-miR-128a boosted the effect of pembrolizumab on laryngeal cancer cells, perhaps via the p53 pathway. Therefore, hsa-miR-128a might be a novel target in laryngeal cancer treatment.

## 1. Introduction

Head and neck squamous cell carcinomas (HNSCCs) are the sixth most common cancer in the United States, with an estimated 65,410 new cases and 14,620 deaths in 2019 [1]. HNSCCs encompass cancers generated from oral cavity, oropharynx, nasopharynx, hypopharynx, larynx, and sinus. Significantly, laryngeal squamous cell carcinoma is among the most malignant cancers and accounts for 1%–2.5% of all malignancies [2], while limited-stage HNSCCs are often curable with surgical resection or definitive radiotherapy and chemotherapy, such as platinum-based regimens, recurrent, and metastatic HNSCCs are associated with poor prognosis, with a 1-year survival rate of approximately 50% [3]. Indeed, the 5-year overall survival rate of laryngeal cancer is less than 60% [4]. Recently, researchers have better elucidated the molecular and biological characteristics of HNSCCs, developed antiepidermal growth factor receptor therapies like cetuximab, and incorporated these approaches into the treatment guidelines for HNSCCs. However, in cases of advanced stage or recurrent tumors, neither traditional chemotherapy nor targeted therapy can improve prognosis; so, researchers must seek novel approaches.

Recently, immunotherapy has shown promise as a new cancer treatment. It is worth noting that therapies subverting immune checkpoint signals, such as programmed cell death protein 1 (PD-1), have revolutionized the management of cancers [5]. As regards HNSCCs, researches focusing on checkpoint immunotherapies that target the PD-1 signaling pathway are also ongoing. Antibodies inhibiting PD-1 have been approved for the second-line treatment of recurrent or metastatic HNSCCs [6, 7]. Specifically, pembrolizumab is a humanized IgG4 kappa isotype antibody that inhibits the binding of PD-1 with its ligands PD-L1 and PD-L2 [8]. Binding of IgGs can induce antibody-dependent cytotoxicity, leading to the undesired elimination of effector T cells. The IgG4 framework was selected in this treatment because it has reduced binding to low-affinity Fc receptors and does not activate the complement pathway [9, 10]. Pembrolizumab is highly selective for PD-1, with picomolar affinity (Kd: 29 pM) and picomolar antagonism of PD-L1/PD-L2 binding (IC50: 500–1000 pM) [11]. PD-1 antibody clones show significant, dose-dependent tumor growth restriction [8]. In patients with melanoma and non-small-cell lung cancers, it has demonstrated clinical safety and efficacy at dosages between 2 and 10 mg/kg every 3 weeks [12]. A more recent study showed that PD-L1 is regulated by the p53/miR-34/PD-L1 axis in lung cancer [13]. However, the relationship between microRNA and the tumor immune system in laryngeal squamous cell carcinoma has not been investigated. In our previous study, we discovered that BMI-1 regulated p53 in laryngeal squamous cell carcinoma [14], and that the expression levels of hsa-miR-128a showed a negative correlation with those of BMI-1 [15]. We carried out the present study to ascertain the possible mechanisms of action of these relationships. To this end, we performed gene upregulation studies, immunotherapy assay, dual luciferase assay, and immunoprecipitation assay to reveal (1) the relationship between hsa-miR-128a and the p53 pathway in laryngeal squamous cell carcinoma and (2) the effect of hsa-miR-128a upregulation on the pembrolizumab sensitivity of laryngeal cancer cells.

## 2. Materials and Methods

### 2.1. Cell Culture

Hep-2 and AMC-HN8 cell lines are the most frequently used laryngeal squamous cell carcinoma cell lines; thus, they were cultured in the present study and utilized in a series of experiments. After being properly resuscitated, they were cultured with Roswell Park Memorial Institute (RPMI)-1640 medium (GIBCO, Invitrogen, Carlsbad, CA, USA), supplemented with 10% fetal bovine serum (FBS; GIBCO) and incubated in a humidified incubator at 37°C with 5% CO_2_. The culture medium was changed every other day, and the cells were digested with trypsin-EDTA solution (GIBCO) for passaging every 3 days.

### 2.2. Quantitative Real-Time Polymerase Chain Reaction (qRT-PCR)

To evaluate the expression levels of hsa-miR-128a and the genes of the p53 pathway, qRT-PCR was performed using standard protocols. First, the total RNA was extracted; to this end, 1 mL of TRIzol and 100 *μ*L of absolute ethanol were added to the culture plate and left overnight at -20°C to allow RNA sedimentation. The cells were then centrifuged for 10 min at 12,000 rpm at 4°C. The supernatant was pipetted out, and the residue was rinsed using 75% ethanol and centrifuged for 5 min at 7,500 rpm at 4°C. The sediment was then dissolved using DEPC-ddH_2_O, and a 1 *μ*L RNA sample was quantified. Second, to produce cDNA, RNA reverse transcriptase was added to the mixture according to the protocol provided by the manufacturer in the M-MLV1 RT-PCR kit (Promega, Madison, WI). The annealing mixture was formulated using 1 *μ*L of Oligo dT (0.5 *μ*g/*μ*L) and 2 *μ*g of total RNA in RNase-free H_2_O. Bathed the sample warmly for 10 min at 70°C and transferred into ice-water mixture and underwent ice bathing for 10 min. During this period, the template annealed to the Oligo dT. The reverse transcription reaction solution contained 0.5 *μ*L RNasin (Axygen), 2 *μ*L of 10-mM dNTPs (Promega), 4 *μ*L of 5× RT buffer, 1 *μ*L of M-MLV-RTase (Promega), 1 *μ*L of random hexamers (Qiagen, Hamburg, Germany), and 2.5 *μ*L of DEPC H_2_O (Axygen). After incubation for 1 hour at 42°C and then 10 min at 80°C, the cDNA product was produced. Third, a 20 *μ*L reaction mixture was prepared, containing 6 *μ*L of ddH_2_O, 10 *μ*L of SYBR Green Master Mix, 1 *μ*L of a 10 *μ*M forward primer of the target gene, 1 *μ*L of 10 *μ*M reverse primer of the target gene, and 2 *μ*L of stored cDNA solution. In accordance with the manufacturer's protocol, the reaction was run at 95°C for 2 min, followed by 40 cycles of 95°C for 15 s, and one final cycle at 55°C for 1 min. The 2^-⊿Ct^ formula was utilized to calculate the gene expression. In the qRT-PCR, the primer sets (5′-3′) used were as follows: hsa-miR-128a, TATAGGCGCGCCACTGGAGTCAATGAAAGCAA and CCCCGCTAGCTAAGCAATAGCTTTCACAAATT; BMI-1, AGCTTATCCATTGAATTCTTTGACC and TCCTCCTCATACATGACATCAATC; p53, ATTTGCGTGTGGAGTATTTGGAT and CCCAGGACAGGCACAAACAC; and p16, CTGCGGAGAGGGGGAGAG and CATCATCATGACCTGGATCGG.

### 2.3. Upregulation of Hsa-miR-128a via Lentiviral Transfection

As in our previous research [16], the transfer vector pLenO-RIP was used to transfer the target gene to lentiviruses. Next, hsa-miR-128a was synthesized, which is a mimic hsa-miR-128a that bears the upstream Mlu I and downstream Not I restriction enzyme sites. After enzyme digestion, the lentiviral vector and target sequences were ligated. Using the protocols given in the AxyPrep Plasmid Miniprep Kit (Axygen), the lentiviral plasmids were extracted; then, the hsa-miR-128a lentiviral plasmids were transfected into 293 T cells. Later, the lentiviruses harboring hsa-miR-128a were transfected into laryngeal cancer Hep-2 cells and AMC-HN8 cells. The qRT-PCR was performed to evaluate the interference rate.

### 2.4. Immunotherapy Assay

The Hep-2 and AMC-HN8 cells were cultured in RPMI-1640 with 10% FBS and then transferred to 96-microwell plates with a density of 2 × 10^4^/100 *μ*L. Three groups of each cell line were designed: a wild-type control group, an hsa-miR-128a group, and a red fluorescent protein (RFP) negative control group. The cells were treated with pembrolizumab (Selleck Chemicals, Shanghai, China) with concentrations of 3 *μ*g/mL, 6 *μ*g/mL, and 12 *μ*g/mL, and the treatment duration was either 24 hours or 48 hours. The culture medium containing chemotherapeutics was cleaned out at preestablished time points. Next, 80 *μ*L of RPMI-1640 and 20 *μ*L of 0.5 mg/mL MTT solution were added into each well. The mixed solution was kept in a water bath at 37°C for 4 hours, and then 100 *μ*L of DMSO was added. The solution was vibrated slowly for 10 minutes to adequately dissolve the crystals. Optical density was measured at 490 nm using an enzyme-linked immunosorbent assay microplate reader (Biorad 680). To this end, the following equations were used: survival rate (SR) = (mean absorbance of the test well/mean absorbance of the control) × 100%; inhibition rate = 100% − SR. All experiments were performed three times.

### 2.5. Dual Luciferase Assay

The luciferase assay was performed using the Dual-Luciferase Reporter Assay system (Promega) in accordance with the manufacturer's protocol. The putative hsa-miR-128a target sites from the BMI-1 3′ untranslated region (UTR) were cloned into the 3′ UTR of the *Renilla* luciferase gene. The pLUC-BMI-1-WT vector was used, which contained the 3′ UTR of the *BMI-1* gene. During transfection, the Plasmid Mini Kit (Omega) was used according to the manufacturer's instructions. The diluted plasmids and lipofectamine were fully mixed at room temperature to form a plasmid–lipofectamine compound. Forty-eight hours after transfection, the cell passive lysis buffer (Promega) was added. After complete lysis, the cells were centrifuged for 5 minutes. The relative light units of the 20 *μ*L sample were measured after 100 *μ*L of firefly luciferase was added. Next, 100 *μ*L of *Renilla* luciferase was added to allow a second measurement. Specifically, *Renilla* luciferase activity was normalized to firefly luciferase activity, and the relative luciferase activity was calculated. These luciferase measurements were performed three times. The total luciferase activity was normalized to the *Renilla* luciferase activity and presented in terms of relative activity to the corresponding negative control (assigned a value “1”). Values denote the mean ± standard deviation of three independent assays.

### 2.6. Immunoprecipitation Assay

The laryngeal cancer cells were lysed in a 15 mL tube using 350 *μ*L of 0.5% lysis buffer. The resuspending solution was transferred to a 1.5 mL Eppendorf tube, which was then centrifuged and lysed for 40 minutes. For each immunoprecipitation, 8 *μ*L of mouse BMI-1 antibody (ab14389; Abcam, Cambridge, MA, USA) was added to the supernatant of the lysed samples, and mouse IgG was used as a control. Precleared extracts were incubated with 25 *μ*L protein A/G-agarose beads (Pierce) in lysis buffer containing 0.05% BSA and antibodies under constant shaking at 4°C overnight. After incubation, agarose bead-bound immunocomplexes were rinsed three times with lysis buffer containing 0.25% NP-40. Next, 80 *μ*L of SDS loading buffer was added to the samples and incubated for 5 minutes at 100°C. Western blot was performed following the instructions of manufacturer to evaluate the effects of immunoprecipitation.

### 2.7. Statistical Analysis

All the results are presented as mean ± standard deviation (SD) for at least three independent experiments when two independent samples were compared. Statistical significance was assessed using independent sample *t*-tests. When comparing three independent groups, analysis of variance and Kruskal–Wallis tests was performed. Stata 12.0 (StataCorp LP, College Station, TX, USA) and SPSS version 22.0 (SPSS Inc, Chicago, IL, USA) were used for data processing and statistical comparisons. All *p* values <0.05 were considered statistically significant.

## 3. Results

### 3.1. The Cell Lines of Laryngeal Squamous Cell Carcinoma Overexpressing Hsa-miR-128a Are Constructed and Cultured

The most commonly used cell lines of laryngeal squamous cell carcinoma, Hep-2 cell line, and AMC-HN8 cell line were cultured appropriately according to the instructions. As in our previous research [15], two stable laryngeal cancer cell lines with upregulated hsa-miR-128a were established. The pLenO-RIP transfer vector was used, and the double-stranded target sequences with hsa-miR-128a mimic were inserted into the Not I and MIu I cloning sites. Two groups were established in the present study: the negative control RFP group and the hsa-miR-128a-RFP group which contained both the target plasmid and the fluorescence plasmid. The interference effect was evaluated using qRT-PCR. As Figure 1 shows, the expression of hsa-miR-128a was dramatically increased in both Hep-2 and AMC-HN8 laryngeal cancer cells after transfection of lentiviruses harboring hsa-miR-128a. The constructed cell lines were also cultured in a humidified incubator at 37°C with 5% CO_2._ The culture medium was changed every other day, and the cells were passaged for further experiments.

### 3.2. The Outcomes of Pembrolizumab on Laryngeal Cancer Cells Were Enhanced by Hsa-miR-128a Upregulation

To evaluate the effect of pembrolizumab on laryngeal cancer cells, a chemotherapy assay was performed. The Hep2 and AMC-HN8 laryngeal cancer cells were treated using 3 *μ*g, 6 *μ*g, and 12 *μ*g of pembrolizumab. First, the inhibition rates were evaluated after 24 hours of treatment. As shown in Figure 2(a)i, the inhibition rates in all three groups of Hep2 cells increased with the concentration of immunotherapeutic drug. At each immunotherapeutic concentration, the inhibition rate in Hep2 cells overexpressing hsa-miR-128a was markedly higher than that in the control cells (*p* < 0.05). Extending the treatment duration to 48 hours, the inhibition rates increased in all three groups. At higher immunotherapeutic concentrations, inhibition rates also became higher. Moreover, the inhibition rates in the in Hep2 cell groups overexpressing hsa-miR-128a were significantly higher than the rates seen in two other groups (*p* < 0.05) (Figure 2(a)ii). Second, a chemotherapy assay was performed in AMC-HN8 cells. The cells were also treated with either 3 *μ*g, 6 *μ*g, or 12 *μ*g of pembrolizumab. After 24 hours, the inhibition rates were evaluated. With increasing dosage, the inhibition rates increased in all three groups, and the AMC-HN8 cell group overexpressing hsa-miR-128a had markedly higher inhibition rates than the control groups (*p* < 0.05), as shown in Figure 2(b)i. Prolonging the treatment duration to 48 hours, the inhibition rates showed a dramatic increase, and the group overexpressing hsa-miR-128a had markedly higher inhibition rates than those seen in other groups (*p* < 0.05) (Figure 2(b)ii).

### 3.3. Hsa-miR-128a Confers these Effects via the p53 Pathway

To ascertain the mechanism of action of hsa-miR-128a in laryngeal cancer cells, a dual luciferase assay was performed. As presented in Figure 3, the relationship between hsa-miR-128a and the *BMI-1* gene was investigated. We subjected the wild-type and mutant *BMI-1* genes to the dual luciferase assay and calculated the relative luciferase activities, which differed significantly between the negative control and cells overexpressing hsa-miR-128a (*p* < 0.05) in the case of wild-type *BMI-1*. With mutant *BMI-1*, no significant difference was observed, indicating that hsa-miR-128a conferred its effects by targeting *BMI-1*. This result was confirmed by the immunoprecipitation assay in which the exogenous expression of hsa-miR-128a strongly reduced the amount of the immunoprecipitated BMI-1 protein in AMC-HN8 cells (Figure 4). Since the *BMI-1* gene functions within the p53 pathway, we used qRT-PCR to compare the expression of genes germane to the p53 pathway. In Hep2 cells, when hsa-miR-128a was upregulated, the expression of BMI-1 decreased significantly (*p* < 0.05), while the expression of p53 and p16 increased (*p* < 0.05 in both cases). In AMC-HN8 laryngeal cancer cells, the results were consistent with those in Hep2 cells (Figure 5).

## 4. Discussion

Laryngeal squamous cell carcinoma is one of the most common head and neck malignancies. As understanding of its pathogenesis has increased, comprehensive treatment appears to be increasingly important. Recently, immunotherapy has shown promise as a novel cancer treatment. The discovery of effective immunotherapeutic methods that subvert immune checkpoint signals such as PD-1 has revolutionized the management of cancers, including HNSCCs. However, the mechanisms of immunotherapeutic strategy in laryngeal squamous cell carcinoma have not been investigated. In the present study, an immunotherapy assay was performed to investigate the influence of hsa-miR-128a on pembrolizumab. The laryngeal Hep2 and AMC-HN8 cell lines were used, and the laryngeal cancer cells were divided into three groups: wild-type cells, cells overexpressing hsa-miR-128a, and negative control RFP cells. These three groups were treated using pembrolizumab, and the influences of pembrolizumab concentration as well as hsa-miR-128a expression levels on the inhibition rates were evaluated. We found that the inhibition rates increased with the pembrolizumab concentration in all three groups of Hep2 cells, and that the inhibition rate in the cells overexpressing hsa-miR-128a was markedly higher than those in the control groups. As the treatment duration was increased to 48 hours, the differences in the inhibition rates became more significant. Moreover, when administering pembrolizumab to AMC-HN8 cells, similar results were obtained, indicating that hsa-miR-128a can increase the effect of pembrolizumab on laryngeal cancer cells.

It has been reported that hsa-miR-128a inhibited tumor proliferation by targeting *BMI-1* in prostate cancer [16]; thus, we performed dual luciferase to determine the potential relationship between hsa-miR-128a and *BMI-1* in laryngeal cancer cells. The dual luciferase assay revealed that, in laryngeal cancer, hsa-miR-128a targets the *BMI-1* gene to confer its effect, consistent with Venkataraman's results [17]. In a previous study, we found that *BMI-1* plays a role in the p53 axis; so, hsa-miR-128a may also confer its effect via the p53 pathway. Results of qRT-PCR showed that upregulating the expression of hsa-miR-128a increased the expression of p53 and p16, while it decreased the expression of BMI-1, confirming our hypothesis. These findings indicate a new role for p53 modulation of the tumor immune response in laryngeal cancer by regulating PD-1 through hsa-miR-128a. However, the experiments were performed on two commonly used laryngeal cell lines. Hence, they may not provide a complete understanding of the mechanisms. In our future research, we will perform the further experiments on more laryngeal cancer cell lines to furtherly confirm our conclusions. Furthermore, p53 binds to hsa-miR-34a during apoptosis, DNA damage, and cell cycle [18–20]; thus, further experiments should explore these mechanisms as well.

In conclusion, the present study found that the overexpression of hsa-miR-128a augments the effect of pembrolizumab on laryngeal cancer cells and that hsa-miR-128a targets *BMI-1* to confer this effect. Additionally, we discovered that hsa-miR-128a plays a significant role in the p53 pathway. As such, we identified a novel mechanism by which tumor immune evasion of laryngeal cancer is regulated by the PD-1/hsa-miR-128a/p53 axis, suggesting that hsa-miR-128a-based therapy may be a novel approach for laryngeal cancer treatment.

## Figures and Tables

**Figure 1:** The overexpression of hsa-miR-128a via lentiviral transfection. (a) The qRT-PCR revealed that hsa-miR-128a expression was dramatically increased in Hep-2 cells via lentiviral transfection (^∗^*p* < 0.05). (b) The expression of hsa-miR-128a was significantly increased in AMC-HN8 cells via lentiviral transfection (^∗∗^*p* < 0.01).

**Figure 2:** Hsa-miR-128a influenced the inhibition rate of pembrolizumab on laryngeal cancer cells. (a) The immunotherapy assay was performed on laryngeal cancer Hep2 cells. (i) 3 *μ*g, 6 *μ*g, or 12 *μ*g pembrolizumab was added to Hep2 cells and cultured for 24 hours. The inhibition rate was significantly different among wild-type Hep2 cells, Hep2 cells overexpressing hsa-miR-128a, and negative control RFP cells (*p* < 0.05). (ii) Hep2 cells treated with pembrolizumab were cultured for 48 hours. The inhibition rate differed significantly among the three groups (*p* < 0.05). (b) The immunotherapy assay was performed in AMC-HN8 laryngeal cancer cells. (i) Wild-type AMC-HN8 cells, AMC-HN8 cells overexpressing hsa-miR-128a, and negative control RFP cells were treated using either 3 *μ*g, 6 *μ*g, or 12 *μ*g of pembrolizumab and incubated for 24 hours. The group with higher expression levels of hsa-miR-128a had markedly higher inhibition rate than those in the other two groups (*p* < 0.05). (ii) The three groups of cells were incubated with pembrolizumab for 48 hours, and the inhibition rates of AMC-HN8 cell group overexpressing hsa-miR-128a were significantly higher than those in the other two groups (*p* < 0.05).

**Figure 3:** *BMI-1* is a target of hsa-miR-128a confirmed by dual luciferase assays. (a) Sequences were compared between mature hsa-miR-128a and the wild-type (WT) and mutant (MUT) target sites in the 3′ UTR of BMI-1. (b) Cells were cotransfected with pMIR-REPORT containing the empty control, wild-type, or mutant target site of the BMI-1 3′ UTR plus hsa-miR-128a or negative control mimic for 48 hours. The luciferase activities were normalized to *Renilla* luciferase activity and presented as relative activities to the corresponding negative control. Values were calculated from three independent assays (^∗^*p* < 0.05).

**Figure 4:** Hsa-miR-128a targeted BMI-1, as shown by Western blot analysis of BMI-1 protein after immunoprecipitation-mediated enrichment in laryngeal AMC-HN8 cells transfected with hsa-miR-128a mimics or control for 48 hours. The exogenous expression of hsa-miR-128a strongly reduced the amount of immunoprecipitated BMI-1 protein in AMC-HN8 cells.

**Figure 5:** The expression of hsa-miR-128a influenced the p53 pathway. The qRT-PCR was used to evaluate the expression levels of representative genes of the p53 pathway. (a) In Hep2 cells, when upregulating hsa-miR-128a, the expression levels of BMI-1 decreased significantly (^∗^*p* < 0.05), and the expression levels of p53 and p16 increased dramatically (^∗∗^*p* < 0.01, ^∗∗∗^*p* < 0.001). (b) In AMC-HN8 laryngeal cancer cells, overexpressing miR-128a caused reduced BMI-1 expression (^∗^*p* < 0.05) and higher expression of p53 and p16 (^∗∗^*p* < 0.01, ^∗∗∗^*p* < 0.001).

## Data Availability

The data used to support the findings of this study are available from the corresponding author upon request.

## References

[1] Siegel R. L., Miller K. D., Jemal A. (2019). Cancer statistics, 2019. *CA: a Cancer Journal for Clinicians*.

[2] Bai Y., Shao Y., Li H., Xue W., Quan F., Wu S. (2016). Ki-67 is overexpressed in human laryngeal carcinoma and contributes to the proliferation of Hep2 cells. *Oncology Letters*.

[3] Vermorken J. B., Mesia R., Rivera F. (2008). Platinum-based chemotherapy plus cetuximab in head and neck cancer. *The New England Journal of Medicine*.

[4] Markou K., Christoforidou A., Karasmanis I. (2013). Laryngeal cancer: epidemiological data from *Ν*orthern Greece and review of the literature. *Hippokratia*.

[5] Ribas A., Wolchok J. D. (2018). Cancer immunotherapy using checkpoint blockade. *Science*.

[6] Cohen E. E. W., Soulières D., le Tourneau C. (2019). Pembrolizumab versus methotrexate, docetaxel, or cetuximab for recurrent or metastatic head-and-neck squamous cell carcinoma (KEYNOTE-040): a randomised, open-label, phase 3 study. *Lancet*.

[7] Ferris R. L., Blumenschein G., Fayette J. (2016). Nivolumab for recurrent squamous-cell carcinoma of the head and neck. *The New England Journal of Medicine*.

[8] Patnaik A., Kang S. P., Rasco D. (2015). Phase I study of pembrolizumab (MK-3475; anti-PD-1 monoclonal antibody) in patients with advanced solid tumors. *Clinical Cancer Research*.

[9] Tao M. H., Canfield S. M., Morrison S. L. (1991). The differential ability of human IgG1 and IgG4 to activate complement is determined by the COOH-terminal sequence of the CH2 domain. *The Journal of Experimental Medicine*.

[10] Scapin G., Yang X., Prosise W. W. (2015). Structure of full-length human anti-PD1 therapeutic IgG4 antibody pembrolizumab. *Nature Structural & Molecular Biology*.

[11] Ahamadi M., Freshwater T., Prohn M. (2017). Model-based characterization of the pharmacokinetics of pembrolizumab: a humanized anti-PD-1 monoclonal antibody in advanced solid tumors. *CPT: Pharmacometrics & Systems Pharmacology*.

[12] Garon E. B., Rizvi N. A., Hui R. (2015). Pembrolizumab for the treatment of non-small-cell lung cancer. *The New England Journal of Medicine*.

[13] Cortez M. A., Ivan C., Valdecanas D. (2015). PDL1 regulation by p53 via miR-34. *JNCI: Journal of the National Cancer Institute*.

[14] Chen H., Zhou L., Dou T., Wan G., Tang H., Tian J. (2011). BMI1's maintenance of the proliferative capacity of laryngeal cancer stem cells. *Head & Neck*.

[15] Chen H., Jin L., Zhou L., Huang J. M. (2018). Overexpressed miR-128a enhances chemoradiotherapy to laryngeal cancer cells and its correlation with BMI1. *Future Oncology*.

[16] Jin M., Zhang T., Liu C. (2014). miRNA-128 suppresses prostate cancer by inhibiting BMI-1 to inhibit tumor-initiating cells. *Cancer Research*.

[17] Venkataraman S., Alimova I., Fan R., Harris P., Foreman N., Vibhakar R. (2010). MicroRNA 128a increases intracellular ROS level by targeting Bmi-1 and inhibits medulloblastoma cancer cell growth by promoting senescence. *PLoS One*.

[18] He L., He X., Lim L. P. (2007). A microRNA component of the p53 tumour suppressor network. *Nature*.

[19] Chang T. C., Wentzel E. A., Kent O. A. (2007). Transactivation of miR-34a by p53 broadly influences gene expression and promotes apoptosis. *Molecular Cell*.

[20] Tarasov V., Jung P., Verdoodt B. (2007). Differential regulation of microRNAs by p53 revealed by massively parallel sequencing: miR-34a is a p53 target that induces apoptosis and G1-arrest. *Cell Cycle*.

